# DPP-4 Inhibitor Improved the Cognitive Function in Diabetic Rats

**DOI:** 10.1155/2022/8280389

**Published:** 2022-11-18

**Authors:** Ying Hu, Jiancheng Wang, Jiao Wang, Wen Chen, Qin Zhang

**Affiliations:** ^1^Department of Endocrinology and Metabolism, First Affiliated Hospital of Nanchang University, Nanchang, Jiangxi 330006, China; ^2^Jiangxi Clinical Research Center for Endocrine and Metabolic Disease, Nanchang, Jiangxi 330006, China; ^3^Jiangxi Branch of National Clinical Research Center for Metabolic Disease, Nanchang, Jiangxi 330006, China; ^4^Department of Anesthesiology, First Affiliated Hospital of Nanchang University, Nanchang 330006, Jiangxi Province, China

## Abstract

Diabetes-associated cognitive dysfunction is a major problem of the international community. Dipeptidyl peptidase-4 (DPP-4) inhibitors are drugs with hypoglycemic effect widely used in diabetic treatment in clinic. In this article, we studied the effect of the DPP-4 inhibitor saxagliptin on cognitive function in diabetic rats. Firstly, to observe cognitive dysfunction caused by diabetes, we built the diabetic rat model. Subsequently, the effect of diabetes on cognitive function was evaluated by Morris Water Maze Task. Thirdly, the mechanism of the alleviation effect of DPP-4 inhibitor on cognitive dysfunction was investigated. Specifically, (1) the anti-inflammation mechanism was revealed by quantifying the accumulation of the inflammatory factor interleukin-1*β* (IL-1*β*) in the hippocampus area by western blotting and the glial fibrillary acidic protein (GFAP) by immunohistochemistry; (2) the anti-tau phosphorylation mechanism was revealed by quantifying phosphorylated tau by western blotting. This work represents the first study demonstrating the alleviation effect of DPP-4 inhibitor on cognitive dysfunction caused by diabetes. Results obtained here could be useful to seeking for a medical solution with high efficacy to the diabetes-associated cognitive dysfunction.

## 1. Introduction 

Diabetes is one of the most ubiquitous chronic endocrine diseases in the world. According to the statistic, over 387 million people suffer from diabetes globally, and the incidence of diabetes in adults has reached up to 11.6% of the Chinese nation. It is estimated by 2035, the number of the diabetics in the world will exceed 600 million [1]. Diabetes is frequently accompanied by the incidence of cognitive dysfunction. It is due to the pathological changes in the microvessel caused by diabetes, which could lead to cerebrovascular damage and thus damage the central nervous system [2]. Cognitive dysfunction has many manifestations in clinic, including loss of memory, reduced recognition and understanding ability, and even the complete loss of daily activity [3]. Nevertheless, various complications of diabetes could deteriorate the progress of cognitive dysfunction [4]. The cognitive dysfunction makes the diabetics less able to realize they are sick, which could severely lower their compliance to therapy and diet control and result in the extreme fluctuation of the blood glucose level. The instability of the blood glucose level again deteriorates the cognitive dysfunction in return [5]. In such a vicious cycle, there is hardly a guarantee of full recovery from diabetes. Therefore, the prevention and treatment of the cognitive dysfunction caused by diabetes are of great significance. At present, the most widely used drugs in treating cognitive dysfunction include tacrine, rivastigmine, galanthamine, donepezil, memantine, etc. [6]. These drugs function as precursor of acetylcholine, inhibitor of acetylcholine esterase, and activator of cholinergic receptor, and thus only have the efficacy of temporarily alleviating clinical symptoms [7]. Seeking for an effective medical solution to the cognitive dysfunction, especially the diabetes-associated cognitive dysfunction, remains challenging.

Screening from the available antidiabetic drugs provides as the primary option to discover a specific compound with additional efficacy of improving the patient's cognitive function. Furthermore, investigating the mechanism of its pharmacological function will provide some leads in maintaining intact cognitive function of the diabetics in clinical treatment. Recently, researches have confirmed that the glucagon-like peptide 1 (GLP-1) plays an important role in treating degenerative diseases of the central nervous system such as Alzheimer, Parkinson, and vascular dementia, and thus could improve the patients' cognitive function [8].

In addition, hyper-phosphorylated tau has neurotoxicity, which can induce the neuronal necrosis [9]. Abnormal hyper-phosphorylation of tau affects its physiological function, thereby leads to the formation of neurofibrillary tangles, and consequently accelerates the deterioration of degenerative diseases [10]. Studies have shown inhibiting the hyper-phosphorylation of tau can effectively relieve patients' cognitive dysfunction and has therapeutic effects on Alzheimer's disease and other symptoms [11]. The level of dipeptidyl peptidase-4 (DPP-4) in some diabetic patients is elevated, and it is speculated that dipeptidyl peptidase-4 may be related to fat metabolism in diabetic patients [12]. The use of DPP-4 inhibitors can improve glycemic control in patients with type 2 diabetes [13]. The dipeptidyl peptidase-4 (DPP-4) inhibitors are new antidiabetic drugs which are effective in increasing endogenous GLP-1 availability [14, 15]. A variety of DPP-4 inhibitors have been widely used in the treatment of diabetes, among which the effect of saxagliptin on blood glucose control is higher than other oral hypoglycemic drugs [14, 16]. However, it remains unknown whether DPP-4 inhibitors are functional in treating diabetes-associated cognitive dysfunction.

Thus, in this work, we investigated the effect of the DPP-4 inhibitor saxagliptin on improving cognitive function in diabetic rats. Furthermore, we evaluated its efficacy in reducing inflammation and tau hyper-phosphorylation in the hippocampus of diabetic rats. The mechanism of the medical function of saxagliptin was finally discussed. The results obtained here provide information for the discovery and development of highly effective drugs to diabetes-associated cognitive dysfunction.

## 2. Materials and Methods

### 2.1. Animals

This study was performed in accordance with regulations for the Care and Use of Laboratory Animals and approved by the Animal Ethics Committee of Nanchang University. Forty-two adult healthy male Sprague-Dawley rats (160–200 g) used in this study were obtained from the Laboratory Animal Center of Nanchang University.

All the rats were bred under standard conditions (20–24°C, 55% ± 5% relative humidity, and 12-h/12-h dark/light cycle) with free access to food and water. All the rats were acclimated to laboratory conditions for 1 week prior to the experiment. At the beginning of the experiment, the rats were randomly divided into normal control group (NC, *n* = 14) and diabetic modeling group (*n* = 28). Rats in the NC group were fed with normal diet, while rats in the diabetic modeling group were fed with high sugar and high fat diet (composition: 67.5% normal feeds, 20% sucrose, 10% pig oil, and 2.5% powder of yolk). After 4 weeks of feeding, rats in the diabetic modeling group were fasted for 12 h but allowed free access to water, then injected with streptozotocin (STZ) intraperitoneally at a dose of 30 mg/kg (currently available, appropriate amount of STZ in the dark, 0.1 mol/L citric acid-sodium citrate in the buffer ice bath, pH = 4.4). 72 h after injection, rats with fasting blood glucose ≥16.7 mmol/L were randomly divided into diabetic model group (DM, *n* = 12) and DPP-4 inhibitor treatment group (DM-S, *n* = 12). Rats in the NC group were weighed and given corresponding dose of citric acid-sodium citrate buffer intraperitoneally instead of  STZ. The DM-S group was given saxagliptin by intragastric administration at a dose of 10 mg/Kg/d for 12 weeks, while the NC group and the DM group were given an equal volume of normal saline in the same manner.

### 2.2. Morris Water Maze Task

24 h after treatment with DPP-4 inhibitor, rats were subjected to the Morris Water Maze (MWM) test to evaluate the learning and memorizing abilities. A round, black painted pool (diameter, 180 cm; depth, 50 cm) was filled with water to a depth of 30 cm and the water was made opaque by the addition of black nontoxic ink. The water temperature was maintained at 24 ± 1°C. The pool was divided into four quadrants and a platform (diameter, 10 cm) was submerged approximately 2 cm below the water line in the center of one quadrant. Trials were started at 9 a.m. by releasing the rat into the water facing the outer edge of the pool at one of the quadrants (in a random sequence) and letting the rat escape to the submerged platform. Once the rat arrived at the platform, it was allowed to stay on it for 30 s. The rat was allowed to swim for a maximum time of 60 s in a trial. The time it spent in reaching the platform was defined as escape latency. Both the escape latency and the swimming distance were recorded. If the rat failed to get the platform within 60 s, it was manually guided to the platform and allowed to stay on it for 30 s and the escape latency was recorded as 60 s. All the tested rats received four training trials a day for 5 consecutive days, with 10- to 15-min interval between trials. On the sixth day, the platform was removed, and each rat was allowed to swim freely for 60 s. The number of times that the rat crossed over the previous platform site, the swimming distance, and swimming time in the target quadrant were all recorded and analyzed. Each rat's swimming path was tracked by a computerized video system (Electric factory of Anhui, China).

### 2.3. Measurement of Blood Glucose

Blood samples were collected from rats before and after treatment with DPP-4 inhibitor. The blood glucose level was measured using 3-uL drop of blood obtained by nicking the tail vein and a One Touch Ultra Link Blood Glucose Meter (Life Scan, Shanghai, China).

### 2.4. Tissue Preparation

After the MWM test, all rats were sacrificed by spinal dislocation. The brains from each group were harvested and the hippocampus was isolated from brain in the ice. The left half of the hippocampus placed in cryopreservation tube was frozen immediately in liquid nitrogen and then stored at −80°C for total protein extraction. Meanwhile, the right hippocampus was fixed in 10% formaldehyde, embedded in paraffin and coronally sectioned (4 *μ*m) for hematoxylin-eosin (HE) staining.

### 2.5. HE Staining

Before immunostaining, 4-um-thick tissue sections were dewaxed in xylene and fixed on poly-L-lysine-coated slides. The tissue sections were dewaxed by xylene and gradient ethanol and stained with hematoxylin (Beyotime, Shanghai) for 3 min. It was differentiated with 1% ethyl alcohol hydrochloride for 30 s, then dyed with 0.5% eosin for 3 min, then dehydrated with gradient ethanol and xylene successively. After drying in a fume hood, the sheet was sealed with neutral gum. Neuronal damage in the hippocampus was analyzed at 400 × magnification (Nikon, Japan).

### 2.6. Immunohistochemistry

After MWM experiment and blood glucose measurement, six rats were randomly selected from each group and anesthetized by intraperitoneal injection of 0.5% sodium pentobarbital at a dose of 50 mg/kg. Their hearts were rapidly exposed, and an infusion needle was inserted into the ascending aorta via the left ventricular and infused with 200 ml of heparin saline (12.5 U/ml) rapidly until effluent liquid from the right atrial appendage was colorless and transparent. 4% paraformaldehyde fixative solution was reperfused slowly for about 30 min. Then their brains were rapidly removed and placed in fixation at 4°C for overnight. After dehydration in alcohol and xylene, the slices were embedded in paraffin and sectioned (4 *μ*m thick).

Sections were deparaffinized, rehydrated with decreasing strengths of ethanol (100% to 50%), and then incubated with 3% H_2_O_2_ for 15 min at 37°C. Thereafter, brain tissue sections were placed in a 0.01 M citrate buffer, boiled at 95°C for 20 min, then cooled down to room temperature. After being sealed with normal goat serum at 37°C for 15 min, sections were probed with the primary antibody, rabbit anti-rat monoclonal antibody to GFAP (1 : 100, CST, Danvers, MA) overnight at 4°C. Then sections were incubated with the secondary antibody, horseradish peroxidase (HRP)-labeled goat anti-rabbit antibody (BL003A, Biosharp Biotech Co., Ltd., Hefei, China), for 30 min at 37°C. Sections were stained with diaminobenzidine (DAB; P0202; Beyotime Biotech Co., Ltd., Shanghai, China) for 5–10 min under microscope observation, counterstained with hematoxylin for 3 min, and then finally sealed. Five random fields from the CA1, CA3, and DG regions were selected respectively at 400 × magnification. The average optical density of GFAP-positive cells can reflect GFAP expression level and was calculated with Image-Pro Plus 6.0 software (Media Cybernetics, US).

### 2.7. Western Blotting

The hippocampus was harvested, homogenized in RIPA lysis buffer (RIPA: PMSF = 100 : 1) on ice for 15 min, and then centrifuged at 12,000 × *g* for 15 min at 4°C. The supernatant was collected and stored at -80°C. The total protein concentration was quantified by the BCA Protein Assay kit (Beyotime Institute of Biotechnology, China) following the manufacturer's instructions. 100 *μ*g of protein per line was separated using 10% SDS-PAGE and then transferred to PVDF membranes (Millipore Co., Billerica, MA, USA). After blocking with 5% skim milk for 2 h, the membranes were incubated with primary antibodies overnight at 4°C.

The primary antibodies used in this study were as follows: anti-*β*-actin (1 : 1000; CST), anti-IL-1*β* (1 : 1000; CST), anti-tau (1 : 1000; CST), anti-p-tau (s202) (1 : 1000; CST), and anti-p-tau (s396) (1 : 1000; CST). The membranes were then washed with 1 × TBS/0.1% Tween 20 and then incubated with HRP-conjugated anti-rabbit IgG (secondary antibody, 1 : 3000; CST) or HRP-conjugated anti-mouse IgG (secondary antibody, 1 : 3000; CST) at room temperature for 2 h. Subsequently, membranes were washed with 1 × TBS/0.1% Tween 20 three times. Blots were visualized with an ECL detection kit (Beyotime Biotechnology, Shanghai, China) and analyzed using ImageJ software (National Institutes of Health, NIH).

### 2.8. Statistical Analysis

Results were analyzed using SPSS Statistics 23 software. Significant differences relative to the controls were determined using independent-samples *t*-tests. For multiple group comparisons, one-way ANOVA was used to determine the significant differences. All results were presented as mean ± standard. *P* values < 0.05 were considered to be statistically significant (^*∗*^*P* < 0.05, #*P* < 0.05). Each experiment was repeated three times.

## 3. Results

### 3.1. Diabetes Caused Cognitive Dysfunction in Rats and DPP-4 Inhibitor Alleviated the Symptoms

To observe the effect of diabetes on cognitive function and further investigate the potential effect of DPP-4 inhibitor on diabetic cognitive dysfunction, we built diabetic rat model (see Materials and Methods section) and evaluated the rats' learning and recognition ability by MWM test. Comparative analysis was carried out on rats from three groups: the normal control group (NC), the diabetic model group (DM), and the saxagliptin-treated diabetic model group (DM-S). As shown in Figure 1, within the experimental time of 5 consecutive days, the NC group exhibited clearly patterned swimming path in all trials with an average escape latency of 6.1 s, suggesting conscious activity and unaffected recognition ability. However, rats from the DM group were unable to get to the platform and exhibited abnormal circulated swimming path which tended to be more abnormal with the progressing of the test. It seemed that the more high sugar and high fat diet they had eaten, the more confused they were. The average escape latency of the DM group was 56.5 s, which was 9.3 folds that of the NC group, whereas the daily shuttle times and total distance of the two groups were comparable. Thus, it appeared that DPP-4 treatment caused instant confusion and slight inactivity in the rats but did not cause the loss of cognitive function. As expected, but still astonishingly, the DM group exhibited disordered swimming path, and neither recovery of cognitive function nor effective physical activity was observed all over the experimental time period. It seemed that the diabetic rats were completely disabled, which was a definite demonstration of cognitive dysfunction. However, rats from the DM-S group exhibited obvious partial recovery of cognitive function along with the advance of time. These results demonstrated that diabetes could cause cognitive dysfunction in rats and DPP-4 inhibitor saxagliptin could alleviate such cognitive dysfunction symptoms caused by diabetes.

We evaluated the efficacy of daily intragastric administration of DPP-4 inhibitor saxagliptin in diabetic rats on blood glucose. The time points included the starting date of week 4 (before treatment) and 16 after intragastric administration of saxagliptin or saline. The fasting blood glucose of the NC group rats was lower than 10 mM before and after treatment. On the other hand, daily intragastric administration of saxagliptin significantly alleviated hyperglycemia of the diabetic rats, controlling the fasting blood glucose to ∼7 mM from ∼18 mM after 12 weeks of treatment. As a control, the fasting blood glucose increased from ∼18 mM to ∼24 mM after daily intragastric administration of saline (Figure 2). The preliminary results indicate that DPP-4 inhibitor saxagliptin can ameliorate high blood glucose status.

### 3.2. DPP-4 Inhibitor Prohibited Neuron Apoptosis in the Hippocampus Area of Diabetic Rats

To reveal the possible mechanism of how DPP-4 inhibitor saxagliptin alleviates cognitive dysfunction in the diabetics, we investigated the neuron apoptosis in the hippocampus area of these rats. We observed the morphology and structure of the hippocampus area of these tested rats under optical microscope after HE staining. As shown in Figure 3, significantly increased number of apoptotic cells was observed in the diabetic group (DM) as compared with the control group (NC), with the morphological change in scattering and decomposing, which demonstrated a severely deteriorated apoptotic process. However, the number of apoptotic cells of rats from the diabetic rats treated with DPP-4 inhibitor saxagliptin was comparable to that of the control group again, demonstrating a rescue from the diabetic status.

### 3.3. DPP-4 Inhibitor Reduced Inflammation in the Hippocampus in Diabetic Rats

Glial fibrillary acidic protein (GFAP) is the marker of astrocyte activation in the hippocampus, which could indicate the extent of the central inflammation in the hippocampus. Interleukin-1 (IL-1; sub-type IL-1*β*) is the major inflammatory factor closely related to cognitive function. Since glucagon-like peptide 1 (GLP-1) and its analogs were previously confirmed with an inhibitory effect on the neural inflammation and DPP-4 inhibitor can increase the endogenous GLP-1 availability, we investigated the effect of DPP-4 inhibitor on neural inflammation in diabetic rats to further reveal the mechanism of its protective effect on cognitive function damaged by diabetes. The expression level of GFAP in the CA1, CA2, and DG regions of the brain was detected by immunohistochemistry. The level of inflammatory factor, IL-1*β*, in the hippocampus area of these rats was tested by the method of western blotting. As shown in Figure 4, a GFAP expression was increased by about 7 folds in rats from the diabetic group than in those from the NC group. However, the GFAP expression sharply decreased by half in the DM-S group compared with the DM group. As for IL-1*β* (Figure 5), increased IL-1*β* was detected in the DM group rats relative to the NC group. Whereas an obvious reduction in IL-1*β* accumulation was observed in rats from the DM-S group as in those from the DM group. These results suggested that diabetes could trigger inflammation and DPP-4 inhibitor could have an anti-inflammation effect on diabetic rats.

### 3.4. DPP-4 Inhibitor Reduced Tau Hyper-Phosphorylation in the Hippocampus

Hyper-phosphorylated tau has neurotoxicity which can induce the neuronal necrosis. Abnormal hyper-phosphorylation of tau affects its physiological function, thereby leads to the formation of neurofibrillary tangles and consequently accelerates the deterioration of degenerative diseases. We assume hyper-phosphorylation of tau might also be a factor in the incidence of cognitive dysfunction, thus we quantified hyper-phosphorylated tau by western blotting. As shown in Figure 5, the expression of the two forms of phosphorylated tau was abnormally high in rats from the diabetic group. DPP-4 inhibitor treatment has a reducing effect on phosphorylation of tau; however, the level of phosphorylated tau in rats from the DM-S group was still much higher than in those from the NC group.

## 4. Discussion

According to the WHO data, the number of diabetics worldwide is as high as 4.22 billion. Studies have shown that hyperglycemia, insulin resistance, inflammation, oxidative stress, and other factors all will affect cognitive function, so the probability of developing cognitive dysfunction, dementia, and other central nervous system diseases in patients with diabetes is significantly higher than that in normal people, and diabetes is also an independent risk factor for Alzheimer's disease [17, 18]. The cognitive dysfunction caused by diabetes seriously affects the quality of life of patients and their relatives, and greatly increases the burden of social medical care. Therefore, it is of great significance to study the cognitive dysfunction of diabetes.

It is acknowledged that both diabetes and Alzheimer cause cognitive dysfunction through over-activating the central inflammatory system or imbalancing the pro-inflammatory and anti-inflammatory systems, which could cause damage to the neuron [19]. Peripheral inflammatory mediators could directly enter the central nervous system or stimulate microglia and astrocyte in the hippocampus area to secrete inflammatory factors, causing local inflammation and thereby reducing cognition ability [20]. Since diabetes and Alzheimer's disease share many common physiological characteristics, and there are few breakthroughs in the treatment of Alzheimer's disease, many scholars try to use antidiabetics to treat the cognitive impairment of diabetes patients [21]. Clinical studies have found that among the antidiabetics, metformin, insulin, pioglitazone, sitagliptin, and other drugs can significantly improve the cognitive ability of diabetes patients [22].

Dipeptidyl peptidase-4 (DPP-4) inhibitors are a class of new oral antidiabetics for the treatment of type 2 diabetes mellitus (T2DM), which can not only regulate the metabolism of glucose and lipids in vivo, but also improve endothelial function and reduce the pro-oxidation and pro-inflammatory states of injured cells [23]. The clinical use of DPP-4 inhibitors includes vildagliptin, Alogliptin, etc., which has a significant therapeutic effect on diabetes without increasing the risk of infection [14, 24]. Saxagliptin as monotherapy or in combination with metformin reduces the risk of hypoglycemia in patients with type 2 diabetes. Saxagliptin is generally well tolerated in clinical trials, with relatively mild adverse reactions and high safety and efficacy. Therefore, this study chose saxagliptin as the research object to explore the therapeutic effect of saxagliptin, a DPP-4 inhibitor, on diabetes-related cognitive dysfunction.

In this study, a diabetic mouse model was established and treated with saxagliptin intragastric administration. The experimental results showed that the diabetic mice fed with high sugar and high fat had increased blood glucose, lost cognitive function, and swimming path disorder. The cognitive function of mice treated with saxagliptin was partially recovered and hyperglycemia was relieved. To further study the therapeutic mechanism of DPP-4 inhibitors, we examined the hippocampal area of diabetic rats. The results showed that saxagliptin treatment significantly inhibited neuronal apoptosis and the expression of inflammatory factors in the hippocampal area of diabetic mice, suggesting that DPP-4 inhibitor could effectively inhibit the inflammatory response and neuronal apoptosis induced by elevated blood glucose in diabetic mice. The detection of hyper-phosphorylated tau protein showed that the expression of phosphorylated tau protein in the hippocampal area of diabetic mice was abnormally high, while DPP-4 inhibitor treatment could effectively reduce the content of phosphorylated tau protein in mice. The above experimental results indicate that DPP-4 inhibitor can not only control blood glucose in diabetic mice, but also reduce neuronal apoptosis by inhibiting the expression of inflammatory factors and phosphorylated tau protein in the hippocampus of mice, thus improving the cognitive function of mice.

The limitation of this study is that GLP-1 levels in neuro inflammation have not been determined. However, our previous studies have shown that saxagliptin increases the level of active GLP-1 in the brain [25]. In conclusion, the treatment of diabetic mice with saxagliptin can improve hyperglycemia and partially restore cognitive function. DPP-4 inhibitors have therapeutic effects on diabetes-related cognitive dysfunction. This study provides a new idea for antidiabetics in the treatment of diabetes-related cognitive dysfunction and points out a new research direction for the treatment of Alzheimer's disease.

## 5. Conclusion

The results of this study suggest that DPP-4 inhibitors can improve the cognitive function of diabetic rats. After treatment with saxagliptin, the cognitive function of mice was partially recovered and the symptoms of hyperglycemia were relieved, so as to control the blood glucose of diabetic mice. Saxagliptin significantly inhibited the expression of phosphorylated tau protein and inflammatory factor IL-1*β* in hippocampal neurons of diabetic mice and reduced neuronal apoptosis, thus improving the cognitive function of mice.

## Figures and Tables

**Figure 1:** Results of Morris Water Maze Task. (a) The swimming path; (b) the escape latency; (c) the total distance; (d) number of platform crossings; (e) the swimming distance in the target quadrant; and (f) the swimming time in the target quadrant. The shown data represent the average of four parallel physiological replicates. In the experiment for 5 consecutive days, the NC group exhibited clearly patterned swimming path in all trials with an average escape latency of 6.1 s. However, rats from the DM group were unable to get to the platform and exhibited abnormal circulated swimming path. The average escape latency of the DM group was 56.5 s which was 9.3 folds that of the NC group, whereas the daily shuttle times and total distance of the two groups were comparable ^*∗*^*P* < 0.05^*∗∗*^*P* < 0.01.

**Figure 2:** Changes in blood glucose before and after the treatment of rats. The fasting blood glucose of the NC group rats was lower than 10 mM before and after treatment. After daily administration of saxagliptin for 12 weeks in DM-S group, the fasting blood glucose was controlled to ∼7 mM from ∼18 mM. The fasting blood glucose of the DM group increased from ∼18 mM to ∼24 mM after daily intragastric administration of saline. ^*∗*^*P* < 0.05, indicates a significant difference compared with the NC group; #*P* < 0.05 indicates a significant difference compared with the DM group.

**Figure 3:** Morphology and structure of the hippocampus area by HE staining (400 × magnification). The significantly increased number of apoptotic cells was observed in the DM group as compared with the NC group, with the morphological change in scattering and decomposing. However, the number of apoptotic cells of rats from the diabetic rats treated with DPP-4 inhibitors was comparable to that of the NC group again.

**Figure 4:** Effects of DPP-4 inhibitor inflammation in the hippocampus of diabetic rats. (a) Expression of GFAP in CA1, CA2, and DG regions of brain detected by immunohistochemistry (400 × magnification). (b) Quantification of GFAP expression. The GFAP expression was increased by about 7 folds in rats from the DM group than in those from the NC group. However, the GFAP expression sharply decreased by half in the DM-S group compared with the DM group. ^*∗*^*P* < 0.05 indicates a significant difference compared with the NC group; ^*#*^*P* < 0.05 indicates a significant difference compared with the DM group.

**Figure 5:** Western blotting of inflammatory factors and phosphorylated tau protein. The expression of the two forms of phosphorylated tau was abnormally high in rats from the DM group. After treatment with DPP-4 inhibitor, tau phosphorylation expression in DM-S group decreased, but it was still much higher than that in the NC group. As for IL-1*β*, increased IL-1*β* was detected in the DM group rats relative to the NC group. Compared with the NC group, IL-1*β* expression was increased in the DM group. The accumulation of IL-1*β* in DM-S group was significantly lower than that in the DM group.

## Data Availability

The data used to support the findings of the research are included within this article.

## References

[1] Lovic D., Piperidou A., Zografou I., Grassos H., Pittaras A., Manolis A. (2020). The growing epidemic of diabetes mellitus. *Current Vascular Pharmacology*.

[2] Lyu F., Wu D., Wei C., Wu A. (2020). Vascular cognitive impairment and dementia in type 2 diabetes mellitus: an overview. *Life Sciences*.

[3] Mueller K. D., Hermann B., Mecollari J., Turkstra L. S. (2018). Connected speech and language in mild cognitive impairment and Alzheimer’s disease: a review of picture description tasks. *Journal of Clinical and Experimental Neuropsychology*.

[4] Kuo S.-C., Lai S.-W., Hung H.-C. (2015). Association between comorbidities and dementia in diabetes mellitus patients: population-based retrospective cohort study. *Journal of Diabetes and Its Complications*.

[5] Biessels G. J., Despa F. (2018). Cognitive decline and dementia in diabetes mellitus: mechanisms and clinical implications. *Nature Reviews Endocrinology*.

[6] Farooq M. U., Min J., Goshgarian C., Gorelick P. B. (2017). Pharmacotherapy for vascular cognitive impairment. *CNS Drugs*.

[7] Dey A., Hao S., Erion J. R., Wosiski-Kuhn M., Stranahan A. M. (2014). Glucocorticoid sensitization of microglia in a genetic mouse model of obesity and diabetes. *Journal of Neuroimmunology*.

[8] Zhao J., Christian H., Liu K., Li L., Li G. L., Liu Y. (2016). Neuroprotective role of(Val^8)GLP-1-Glu-PAL in an in vitro model of Parkinson’s disease. *Neural Regeneration Research (English version)*.

[9] Ma D.-L., Chen F.-Q., Xu W.-J., Yue W.-Z., Yuan G., Yang Y. (2015). Early intervention with glucagon-like peptide 1 analog liraglutide prevents tau hyperphosphorylation in diabetic db/db mice. *Journal of Neurochemistry*.

[10] Xu W., Yang Y., Yuan G., Zhu W., Ma D., Hu S. (2015). Exendin-4, a glucagon-like peptide-1 receptor agonist, reduces Alzheimer disease-associated tau hyperphosphorylation in the Hippocampus of rats with type 2 diabetes. *Journal of Investigative Medicine*.

[11] Boutajangout A., Wisniewski T. (2014). Tau-based therapeutic approaches for Alzheimer’s disease - a mini-review. *Gerontology*.

[12] Valerio C. M., de Almeida J. S., Moreira R. O. (2017). Dipeptidyl peptidase-4 levels are increased and partially related to body fat distribution in patients with familial partial lipodystrophy type 2. *Diabetology & Metabolic Syndrome*.

[13] Crepaldi G., Carruba M., Comaschi M., Del Prato S., Frajese G., Paolisso G. (2007). Dipeptidyl peptidase 4 (DPP-4) inhibitors and their role in Type 2 diabetes management. *Journal of Endocrinological Investigation*.

[14] Jarvis C. I., Cabrera A., Charron D. (2013). Alogliptin. *The Annals of Pharmacotherapy*.

[15] Rizos E. C., Ntzani E. E., Papanas N. (2013). Combination therapies of DPP4 inhibitors and GLP1 analogues with insulin in type 2 diabetic patients: a systematic review. *Current Vascular Pharmacology*.

[16] Wang M.-M., Lin S., Chen Y.-M. (2015). Saxagliptin is similar in glycaemic variability more effective in metabolic control than acarbose in aged type 2 diabetes inadequately controlled with metformin. *Diabetes Research and Clinical Practice*.

[17] Zilliox L. A., Chadrasekaran K., Kwan J. Y., Russell J. W. (2016 Sep). Diabetes and cognitive impairment. *Current Diabetes Reports*.

[18] Xue M., Xu W., Ou Y.-N. (2019). Diabetes mellitus and risks of cognitive impairment and dementia: a systematic review and meta-analysis of 144 prospective studies. *Ageing Research Reviews*.

[19] Infante-Garcia C., Ramos-Rodriguez J. J., Galindo-Gonzalez L., Garcia-Alloza M. (2016). Long-term central pathology and cognitive impairment are exacerbated in a mixed model of Alzheimer’s disease and type 2 diabetes. *Psych Neuroendocrinology*.

[20] Rosczyk H. A., Sparkman N. L., Johnson R. W. (2008). Neuroinflammation and cognitive function in aged mice following minor surgery. *Experimental Gerontology*.

[21] Muñoz-Jiménez M., Zaarkti A., García-Arnés J. A., García-Casares N. (2020). Antidiabetic drugs in Alzheimer’s disease and mild cognitive impairment: a systematic review. *Dementia and Geriatric Cognitive Disorders*.

[22] Cao B., Rosenblat J. D., Brietzke E. (2018 Oct). Comparative efficacy and acceptability of antidiabetic agents for Alzheimer’s disease and mild cognitive impairment: a systematic review and network meta-analysis. *Diabetes, Obesity and Metabolism*.

[23] Avogaro A., Kreutzenberg S., Fadini G. (2014). Dipeptidyl-peptidase 4 inhibition: linking metabolic control to cardiovascular protection. *Current Pharmaceutical Design*.

[24] van Poppel P. C. M., Gresnigt M. S., Smits P., Netea M. G., Tack C. J. (2014). The dipeptidyl peptidase-4 inhibitor vildagliptin does not affect ex vivo cytokine response and lymphocyte function in patients with type 2 diabetes mellitus. *Diabetes Research and Clinical Practice*.

[25] Kamel N. M., Abd El Fattah M. A., El-Abhar H. S., Abdallah D. M. (2019). Novel repair mechanisms in a renal ischaemia/reperfusion model: s. *European Journal of Pharmacology*.

